# Clinical Efficacy and Safety of Ibuprofen plus Traction, Reposition, and Hip Spica Cast in the Treatment of Developmental Dysplasia of the Hip

This article has been retracted.

**DOI:** 10.1155/2022/1213133

**Published:** 2022-08-09

**Authors:** Dachang Feng, Zhaofa Liu, Haitao Chen, Huanhuan Wang

**Affiliations:** Department of Orthopedics, Foshan Women and Children Hospital, Southern Medical University, No. 11 West Renmin Rd, Foshan 528000, Guangdong, China

## Abstract

**Objective:**

To assess the clinical efficacy and safety of ibuprofen plus traction, reposition, and hip spica cast in the treatment of developmental dysplasia of the hip (DDH).

**Methods:**

Between January 2019 and July 2020, 60 children with DDH treaded in department of orthopedics of our institution were assessed for eligibility and recruited. They were assigned at a ratio of 1 : 1 to receive either traction + reposition + hip spica cast plus analgesia pump (observation group) or traction + reposition + hip spica cast plus analgesia pump and oral ibuprofen (control group). The outcome measures included clinical efficacy, pain scores, unexpected pain calls, the dosage of analgesia pump, and adverse events.

**Results:**

The two groups had similar clinical efficacy (*P* > 0.05). The patients given oral ibuprofen were associated with significantly lower pain scores at 24 h and 72 h postoperatively versus those without oral ibuprofen (*P* < 0.05). Analgesics with oral ibuprofen resulted in fewer unexpected pain calls versus analgesics without oral ibuprofen within 72 h postoperatively (*P* < 0.05). The application of oral ibuprofen in the analgesia pump showed great improvement in lowering the dosage of analgesia pump versus the absence of ibuprofen (*P* < 0.05). The incidence of adverse events was similar between the two groups of patients (*P* > 0.05).

**Conclusion:**

Traction + reposition + hip spica cast plus analgesia pump and oral ibuprofen effectively mitigated postoperative pain in children with DDH and reduces analgesic drug dosage with a high safety profile.

## 1. Introduction

Developmental dysplasia of the hip (DDH) is a serious congenital disorder of the skeletal system that results from developmental malformation of the hip joint due to abnormality of the femoral head to the acetabulum within the joint capsule and is associated with severe pain and dysfunction [1, 2]. The DDH refers specifically to abnormalities in the shape, size, orientation, or histology of the femoral head and acetabulum. It is classified into hip dysplasia, hip subluxation, and hip dislocation according to the severity of the lesion. In China, the DDH has a prevalence of up to 0.08%–0.27%, with a predominance of females. A large body of evidence suggests that better outcomes are associated with a younger age of treatment [3, 4]. Infants and young children are the susceptible population of the disease. At present, conservative abduction braces are the main treatments, of which the Pavlik sling is the most commonly used. Studies have shown that the abduction brace represented by the Pavlik sling has drawbacks, including that the Pavlik sling has a low cure rate for children older than 4 months or Graf IV, which can lead to necrosis of the femoral head, posterior acetabular wall injury, and sciatic nerve and complications such as paralysis or hip dislocation, brachial plexus injury, and skin injury Willey et al. [5].

Traditional Chinese medicine classifies it as “bone arthralgia,” “rheumatic arthralgia,” and “joint running.” “Su Wen·Bi Lun” states “three qi of wind, cold, dampness intermingle, and all the five internal organs would be affected.” Traditional Chinese medicine manipulation can directly act on the muscles and bones of the affected part, which can enhance muscle tension and stability, improve joint movement, local microcirculation, and improve tissue metabolism, exerting good efficacy and safety for conservative treatment of early hip dysplasia [6, 7].

Traction + reposition + hip spica cast is a common clinical treatment for DDH. The osteotomy of the acetabulum and femur frequently required in surgery is frequently associated with intense postoperative pain. Research has demonstrated moderate to severe postoperative pain in approximately 35% of cases and inadequate postoperative analgesia in 70% of cases. The postoperative pain decreases the treatment satisfaction of patients and families and limits postoperative functional recovery, leading to delayed recovery and discharge. The postoperative pain results in a state of stress that suppresses the immune function, and persistent pain inflicts irreversible damage to the physiological functions of the child, which requires timely and effective analgesia [8, 9]. Thus, perioperative analgesic management is of great clinical significance. The clinical difficulties in expression of the severity of pain and the effectiveness of analgesic treatment in children complicate pain assessment and management. The poor progression of analgesic treatment in children is attributed to the high risk of adverse events and toxic reactions to analgesic drugs due to the underdeveloped physiological functions of children [10]. Ibuprofen is a nonsteroidal anti-inflammatory analgesic frequently used for postoperative analgesia in clinical practice. Studies have revealed a similar or improved analgesic effect of ibuprofen combined with or without other analgesics versus other analgesics in adult patients postoperatively. For pediatric and adolescent patients with moderate to severe pain, ibuprofen has also been documented with similar or better analgesic effects [11, 12]. However, postoperative pain relief with ibuprofen for pediatric patients is marginally explored. In accordance, 60 patients with DDH treated in our institution between January 2019 and July 2020 were recruited to assess the clinical efficacy and safety of ibuprofen plus traction + reposition + hip spica cast in the treatment of DDH to provide a clinical reference.

## 2. Materials and Methods

### 2.1. Baseline Data

Before enrollment, the investigators obtained the informed consent from the patients. The protocol was approved by the hospital ethics committee (SH-WU20190102). All procedures were in line with guidelines of the Declaration of Helsinki.

Between January 2019 and July 2020, 60 children with DDH treaded in our institution were assessed for eligibility and recruited. They were assigned (1 : 1) to receive either traction + reposition + hip spica cast plus analgesia pump (observation group) or traction + reposition + hip spica cast plus analgesia pump and oral ibuprofen (control group) (Table 1). Randomization was performed using an online web-based randomizer (http://www.randomizer.org/). For the blindness of the study, randomization procedures and assignments were conducted by independent assistants who were not involved in screening or evaluating participants.

### 2.2. Inclusion and Exclusion Criteria

Inclusion criteria were as follows: children with a clinical diagnosis of developmental dysplasia of the hip, with X-ray manifestations of hip subluxation or complete dislocation, and with traction + reposition + hip spica cast. Exclusion criteria were as follows: children with allergies to opioid analgesics and nonsteroidal drugs, whose parents were not cooperative, and with significant abnormalities in routine examinations and tests on admission.

### 2.3. Methods

Procedure: all children were subjected to skin traction after admission, with an average traction duration of 2–9 days, and the skin traction was released 1 day before surgery. After general anesthesia, the surgeon moved the affected hip to feel the tension of the adductor muscles and performed a trial hip repositioning. The effectiveness of hip repositioning was evaluated intraoperatively by hip arthrography, using an average dose of 1.35 (0.8–1.5) ml of contrast agent Uvexan (Bayer Healthcare Guangzhou Branch, Guangzhou, China), with a needle entry point 2 cm below the adductor tendon of the hip joint. The effectiveness of hip repositioning was evaluated by using Bowen's standard chart after imaging: the proximal femoral epiphysis was below the Hilgenreiner line (H line), 2/3 of the horizontal radius of the femoral head was within the Perkin line, and the femoral head was located below the outer edge of the glenoid hip after repositioning. In the case of unsuccessful repositioning or poor repositioning suggested by hip arthrography, simple incisional repositioning was performed through a small anterior incision. A 2-3 cm surgical incision was made 1-2 cm below the anterior superior iliac spine in the direction of the dermatome, the subcutaneous tissues were separated to the deep fascia, accessed along the space between the broad fascial tensor and sutures, the rectus femoris muscle was cut at the anterior inferior iliac spine and reflexed to expose the joint capsule, the iliopsoas tendon was cut, and the joint capsule was incised obliquely from superior to inferior to the transverse acetabular ligament. The intraarticular fatty tissue and round ligaments were removed, the hip joint was repositioned by flexion and abduction, and the joint capsule was sutured. The rectus femoris muscle was reconstructed and the incision was closed layer by layer. All procedures were performed by 2 senior surgeons. Postoperatively, all cases were immobilized in a hip spica cast after successful repositioning for 5–14 weeks. The hip spica brace was worn all day for 14 weeks after removal of the hip spica cast and then changed to half-day wear until 1 year [13].

On the basis of the treatment of the two groups, modified Gancao Fuzi decoction was given: cassia twig 20 g, Paofu tablet 10 g (fried first), *Atractylodes* 10 g, and honey-fried licorice root 10 g. It was added or subtracted according to the symptoms; for those with severe pain, red peony 10 g and salvia 10 g were added; for those with yin deficiency and fire, *Dendrobium* 10 g and *Ophiopogon japonicus* 15 g were added; for those with qi deficiency, 10 g of *Astragalus* and 10 g of *Codonopsis* were added. The abovementioned traditional Chinese medicines are uniformly decocted by the decoction room of the hospital, one dose per day; it is decocted in 400 ml of water and taken twice in the morning and evening. The course of treatment is 4 weeks.

### 2.4. Outcome Measures

① Clinical efficacy: Excellent: the function and shape of the affected part were completely restored with anatomical repositioning or close to anatomical repositioning. Good: the functional repositioning was achieved, and the function and shape were basically restored. Poor: the function repositioning was failed, with obvious deformity in shape and significantly compromised function. Total clinical efficacy = (excellent + good)/total number of cases × 100%. ② Pain score: Children's Hospital of Eastern Ontario Pain Scale (CHEOPS) was used for pain assessment: the total score was 10 points, with 0–3 points for no pain or mild pain, 4–7 points for moderate pain, and 8–10 points for severe pain. Higher scores indicated more intense pain. ③ Unexpected pain calls: the number of unexpected pain calls was recorded for both groups within 72 h after surgery. ④ Analgesia pump dosage: the analgesia pump was removed at 48 h postoperatively in both groups, and the dosage of analgesia pump medication was recorded by our medical staff after removal. ⑤ Adverse events: the adverse events that occurred during treatment were recorded including vomiting, urinary retention, and respiratory depression.

### 2.5. Statistical Analysis

SPSS 22.0 was used for data analyses, and GraphPad Prism 8 was used for image rendering. The measurement data were expressed as ($\bar{x}\pm s$) and processed using the independent sample *t*-test. Normally distributed measurement data are represented by mean plus and minus standard deviation ($\bar{x}\pm s$); the mean comparison between the two groups was first performed by the F-test for homogeneity of variance, the independent samples *t*-test for homogeneity of variance, and the independent samples *t*-test for heterogeneity of variance; the paired samples *t*-test was used for comparison within the group before and after treatment. The count data were expressed as the number of cases (rate) and analysed using the chi-square test. Differences were considered statistically significant at *P* < 0.05.

## 3. Results

### 3.1. Clinical Efficacy

The two groups had similar clinical efficacy (*P* > 0.05) (Table 2).

### 3.2. Pain Scores

The patients given oral ibuprofen were associated with significantly lower pain scores at 24 h and 72 h postoperatively versus those without oral ibuprofen (*P* < 0.05) (Figure 1).

### 3.3. Unexpected Pain Calls

Analgesics with oral ibuprofen resulted in fewer unexpected pain calls versus analgesics without oral ibuprofen within 72 h postoperatively (*P* < 0.05) (Figure 2).

### 3.4. Dosage of Analgesia Pump

The application of oral ibuprofen in the analgesia pump showed great improvement in lowering the dosage of analgesia pump versus the absence of ibuprofen (*P* < 0.05) (Figure 3).

### 3.5. Incidence of Adverse Events

The incidence of adverse events was similar between the two groups of patients (*P* > 0.05) (Table 3).

## 4. Discussion

The pathological changes of DDH involve structures such as the acetabulum, femoral head, joint capsule, surrounding muscles, and ligaments, and the specific pathogenesis remains yet unclear. Studies have shown that the traditional swaddling position forces the baby's hip joint to be in a straight position, which makes the acetabulum and femoral head mismatch during the development of the acetabulum and eventually progresses to DDH. Another study shows that some women need to use relaxin to relax the pelvic ligaments during childbirth, but relaxin can enter the fetus through the placental barrier, which may lead to relaxation of the ligaments around the acetabulum and become a potential risk of DDH in infants and young children. Adductor tension contracture is an important pathological change in children with DDH aged 0–6 months, and most hips can be reduced after release of the adductor muscle [14, 15].

The prevalence of developmental dysplasia of the hip varies between different geographic regions and races, and the prevalence in China is about 1–3 per 1,000, with the incidence in girls being about 3–6 times higher than that in boys [16]. Currently, multiple factors such as the child's body mass, breech pregnancy, foot deformity, family history of hip dysplasia, and skeletal muscle deformity are considered to be strongly associated with the development of hip dysplasia. Children with congenital dysplasia benefit from early diagnosis and reasonable treatment to achieve a favorable prognosis [17, 18], but there are still some cases with delayed diagnosis or poor conservative treatment efficacy that require surgical treatment. Surgical treatment is mainly to restore the concentric relationship between the femoral head and the acetabulum, whilst avoiding femoral head necrosis and reoperation [19, 20]. Traction + reposition + hip spica cast is a common clinical treatment for DDH. Traction is simple, effective, and time-efficient [21], repositioning aids in the hip repair and restoration [22], and hip spica cast contributes to the recovery of the child's organism and shortens the hospital stay with lower costs [23, 24].

The related pathological changes of hip dislocation are mentioned in the literature of traditional Chinese medicine, and DDH is called “hipbone displacement.” “The Essentials of the Bone-Setting Heart Method” states “for people with hip bone displacement, the buttocks would move obliquely,” which points out the clinical characteristics of hip dislocation. “Prescriptions for Universal Relief” proposed to judge whether hip dislocation occurs by comparing the length of both the lower limbs.

Intraoperative osteotomies of the acetabulum and femur are associated with intense postoperative pain, which inhibits the body's immune function and elicits irreversible damage. Therefore, perioperative analgesic treatment is of great clinical importance. In the choice of the analgesic method, it has been found that single analgesic methods are insufficient for satisfactory results, which are attributable to the inadequacy of pharmacological analgesia by one mechanism of action alone to deal with postoperative pain originating from different signaling pathways transduction. Ibuprofen inhibits cyclooxygenase and reduces the synthesis of prostaglandins and activation of peripheral receptors to exert analgesic and anti-inflammatory effects, but it is prone to platelet inhibition and other adverse reactions. Analgesia pump drugs are opioids that bind to *μ* receptors in the brain and *K* receptors in the spinal cord to achieve analgesia, but they may generate adverse events such as respiratory depression, nausea and vomiting, urinary retention, and drug dependence in children, especially in pediatric patients with immature liver enzyme systems, resulting in difficulties in the clinical selection of drug doses [25, 26]. The combination of these two drugs may provide a complementary and synergistic effect, resulting in optimal analgesia for pediatric patients.

Here, the eligible patients given oral ibuprofen were associated with significantly lower pain scores at 24 h and 72 h postoperatively and fewer unexpected pain calls within 72 h, postoperatively versus those without oral ibuprofen, suggesting that the combined ibuprofen analgesia was effective in mitigating the pain of the children and reducing the number of severe pain episodes. Moreover, the application of oral ibuprofen in the analgesia pump showed great improvement in lowering the dosage of the analgesia pump versus the absence of ibuprofen, indicating that ibuprofen can effectively reduce the amount of opioid medication to attenuate the damage to the children. Furthermore, the similar incidence of adverse events between the two groups herein highlighted the safety profile of ibuprofen in postoperative analgesia.

To sum up, traction + reposition + hip spica cast plus analgesia pump and oral ibuprofen effectively mitigated postoperative pain in children with DDH and reduced analgesic drug dosage with a high safety profile.

## Figures and Tables

**Figure 1:** Comparison of pain scores ($\bar{x}\pm s$). The patients given oral ibuprofen were associated with significantly lower pain scores at 24 h and 72 h postoperatively versus those without oral ibuprofen.

**Figure 2:** Comparison of unexpected pain calls ($\bar{x}\pm s$). Analgesics with oral ibuprofen resulted in fewer unexpected pain calls versus analgesics without oral ibuprofen within 72 h, postoperatively.

**Figure 3:** Comparison of dosage of analgesia pump ($\bar{x}\pm s$). The application of oral ibuprofen in the analgesia pump showed great improvement in lowering the dosage of analgesia pump versus the absence of ibuprofen.

**Table 1:** Comparison of the baseline data (*n* (%)).

	Observation group (*n* = 30)	Control group (*n* = 30)	*t* or *x*^2^	*P* value
Gender			0.073	0.787
Male	11	10		
Female	19	20		
Mean age (year)	7.61 ± 1.41	7.53 ± 1.42	0.219	0.827
Mean body mass (kg)	20.12 ± 3.55	20.24 ± 3.38	−0.134	0.894
Mean height (cm)	110.54 ± 15.73	109.98 ± 15.59	0.138	0.891
Duration of disease (month)	62.72 ± 19.87	62.50 ± 19.71	0.043	0.966

^#^ *P* < 0.05.

**Table 2:** Comparison of clinical efficacy (*n* (%)).

	Observation group (*n* = 30)	Control group (*n* = 30)	*x * ^2^	*P*
Excellent	11	14	—	—
Good	19	16	—	—
Poor	0	0	—	—
Efficacy	30 (100%)	30 (100%)	—	—

^#^ *P* < 0.05.

**Table 3:** Comparison of the incidence of adverse events (*n* (%)).

	Observation group (*n* = 30)	Control group (*n* = 30)	*x * ^2^	*P*
Vomiting	3	2	—	—
Urinary retention	2	2	—	—
Respiratory depression	1	1	—	—
Incidence of adverse events	6 (20%)	5 (17%)	0.111	0.739

^#^ *P* < 0.05.

## Data Availability

The data generated or analysed during this study are included within the article.
